# A Two-Phase Mitosis Detection Approach Based on U-Shaped Network

**DOI:** 10.1155/2021/1722652

**Published:** 2021-10-05

**Authors:** Wenjing Lu

**Affiliations:** School of Information Engineering, Harbin University, China

## Abstract

This paper proposes a deep learning-based method for mitosis detection in breast histopathology images. A main problem in mitosis detection is that most of the datasets only have weak labels, i.e., only the coordinates indicating the center of the mitosis region. This makes most of the existing powerful object detection methods hardly be used in mitosis detection. Aiming at solving this problem, this paper firstly applies a CNN-based algorithm to pixelwisely segment the mitosis regions, based on which bounding boxes of mitosis are generated as strong labels. Based on the generated bounding boxes, an object detection network is trained to accomplish mitosis detection. Experimental results show that the proposed method is effective in detecting mitosis, and the accuracies outperform state-of-the-art literatures.

## 1. Introduction

Breast cancer is one of the main threats to woman health and becomes one of the most leading causes of cancer-related death all over the world. Early diagnosis is believed to be an effective way for promoting the prognosis of breast cancer.

Generally, breast cancer can be classified into three levels in histopathology based on the morphological microstructure of cancerous and the normal cells, i.e., well differentiated, poorly differentiated, and intermediate. Classification is important to the diagnosis and prognosis of breast cancer. The most commonly used classification standard is the BRE system proposed by WHO, in which three indications are used to evaluate the differentiation level. The indications are vasculogenesis degree, nuclear atypia, and mitotic counting.

Among the indications, mitotic counting is the most important, which can be described as the number of cells under mitosis in tumer and around areas. In traditional methods, mitotic counting is done by pathologists. Since the nuclei of cells experiencing mitosis are extremely small, therefore, attention should be highly concentrated. Moreover, the morphology of cells under various stages of mitosis is different, and there may exist enormous normal cells which are similar to mitotic cells. Due to these reasons, mitotic counting is a tedious and error-prone task.

In order to reduce the workload of pathologists, many computer algorithms and systems are proposed to automatically detect mitosis. Traditional automatic mitosis detection methods usually extract handcrafted features from breast histopathology images and train a machine learning algorithm and then perform predictions on testing images based on the trained model. The key issue of such methods is the feature definition. Effective features can greatly increase the accuracy of detection, while badly defined features may dramatically influence the accuracy.

Recently, deep learning has attracted the attention of researchers and becomes a new focus of computer vision. Convolutional neural networks (CNNs) are applied to images, and discriminative features are extracted under appropriate loss functions. Compared with traditional learning-based methods, the most notable advantage of CNN-based ones is that no human interventions are needed throughout the whole procedure. In consideration of the superiority of CNNs, many researchers begin to employ CNN-based methods to detect mitosis in breast histopathology images and achieve competent performances.

In this paper, a CNN-based mitosis detection method is proposed. The whole procedure can be separated into two phases. For the first phase, in consideration of the lack of strong labels in current datasets, a U-shaped network is trained over pixellevel-labeled datasets and used to predict bounding boxes on datasets which only have weak labels. In the second phase, the predicted bounding boxes are then taken as strong labels to train a network for mitosis detection. Contributions of this paper can be summarized as follows.

1. A mitosis detection method is proposed aiming at solving the problem of insufficiency of strongly labeled breast histopathology image dataset. We propose to use pixel-wise-labeled datasets to train a segmentation network, and then, strong labels (bounding boxes) can be generated based on the prediction of the segmentation network. Thus, most of the current weakly labeled datasets can be used for mitosis detection network training
2. For mitosis segmentation, a U-shaped network is trained using a pixelwisely labeled dataset. Benefiting from the multiple frequency downsampling and upsampling layers in the network, the ability of segmenting small targets is promoted, which is suitable for the mitosis segmentation task

The rest of this paper will be organized as follows.  Section 2gives a brief literature review of mitosis detection in breast histopathology images.  Section 3 proposes the mitosis detection method with detailed network structure.  Section 4 provides sufficient experiments and comparisons to show the effectiveness of the proposed method, and finally in Section 5, conclusions are drawn.

## 2. Related Works

Most of the traditional mitosis detection methods are based on image features which are manually designed by computer scientists and pathologists. Huang et al. [1] propose an exclusive independent component analysis (XICA) algorithm to detect mitosis. It is based on the fact that the mitotic nucleus is darker; then, it surrenders in color, and a sparse representation-based classifier is used to extract mitosis from candidates. Considering there may be distinct color variations in breast histopathological images, Tashk et al. [2] propose to use texture features for mitosis detection. An object-oriented complete local binary pattern is designed, and the support vector machine (SVM) is used to separate mitosis from background. Khan et al. [3] propose to employ a Gaussian mixture model (GMM) to model the distributions of mitosis pixels and background pixels, and a context-aware postprocessing is used to reduce false negatives. Tek et al. [4] investigate a set of generic features, i.e., color, binary shape-based, Laplacian, and morphological features to represent mitosis regions. The AdaBoost algorithm is then used to detect mitosis. All these methods employ handcrafted image features and a machine learning algorithm to predict whether image pixels belong to the mitosis region or not. However, since mitotic morphology may vary greatly and the collection of tissue sections obtained by different instruments also increases the diversity of the appearances of histopathological images, image features such as color, texture, and intensity may be incompetent to fully represent mitosis. Besides, designing of such features requires rich experiences of computer scientists and pathologists, and therefore, such methods are not so satisfactory for automatic mitosis detection.

Recently, researchers begin to put their focus on CNN-based automatic mitosis detection methods. CNNs construct high-level semantic features from low-level features and obtain competent performances in many areas of computer vision such as classification, segmentation, and object detection [5–9]. Ciresan et al.'s team [10] is one of the earliest researchers who employ CNNs for mitosis detection. In their work, a CNN with sliding window and max pooling is proposed, and they achieved the first place in ICPR2012 mitosis detection competition. Wang et al. [11] propose a mitosis detection method which combines both handcrafted and CNN features. Although the computational load is reduced by incorporating manually designed features, the overall performance is limited due to the disability of handcrafted features in representing mitosis morphology. Veta et al. [12] propose a similar method and obtain the first place in ICPR2013 mitosis detection contest. Chen et al. [13] use a cascaded CNN to detect mitosis by constructing a two-stage deep network. A rough search network is used to search mitosis candidates and a discriminant network to further select mitosis from candidates. Inspired by the residual conception proposed by He et al. [14], Zerhouni et al. [15] propose a wide residual network (WRN) for mitosis detection. Recently, Li et al. [16] employ faster R-CNN [17] as the detector for mitosis detection. However, since the faster R-CNN is designed as a general purpose object detection network, it is hard to get satisfactory performance on mitosis detection task without sufficient training data.

A main difficulty of mitosis detection is that most existing datasets only have weak labels, i.e., only center points of mitotic nucleus are labeled. It is difficult to construct a valid training set to train a powerful detection network based on such labels. At most occasions, it is unavoidably for pathologists to perform a pixel-level or bounding box-level labeling on such datasets, which is a labor-consuming task. Some researchers intend to solve this problem. For example, Li et al. [18], Zerhouni et al. [15], Cai et al. [19], and Yancey [20] crop a square area around the label point as the region of interest. However, since mitosis is often heteromorphic in shape, a large amount of background pixels are included into the cropped area, which influences the detection performance.

## 3. Method

Mitosis detection can be seen as a special case of object detection. In the past few years, along with the successful employment of CNNs, object detection methods, such as R-CNN [21], fast R-CNN [22], faster R-CNN [17], SPP-Net [23], and YOLO [24], achieve reasonable accuracies and efficiencies. However, such general purpose object detection methods are hard to be employed into the mitosis detection task directly. The main reason is that such methods usually need to have a training dataset with labeled bounding boxes indicating regions of interest. In most existing breast histopathology image datasets, mitosis are weakly labeled, i.e., only the coordinates indicating the centers of mitosis regions are labeled. With such weakly labeled samples, a manual labeling is needed to generate bounding boxes in order to employ a detection algorithm.

To solve this problem, this paper proposes to generate bounding boxes for weakly labeled breast histopathology images and construct a mitosis detection method based on object detection networks. Firstly, a U-shaped network is trained using pixel level-labeled dataset, and this network is used for segmenting mitosis. Based on the segmentation and weak labels, bounding boxes of mitosis are generated for training a detection network. Then, the detection network is used to detect mitosis. The whole process is depicted in Figure 1. In this section, the two stages of the proposed method will be described in detail.

### 3.1. Label Generation

CNNs have been successfully used in biomedical image segmentation. Inspired by the U-Net [25] and the multilevel wavelet CNN (MWCNN) [26], a segmentation network is used in this paper to promote the ability of segmenting small targets. The structure of the network is depicted in Figure 2.

As shown in Figure 2, each CNN block is a 4-layered fully convolutional network (FCN) without pooling and takes the discrete wavelet transform (DWT) subband image as the input except the first layer. Low-frequency and high-frequency bands of DWT in CNN help to fully explore all frequency information of the input image, and the inverse wavelet transform (IWT) plays the role of reconstructing subband images into whole. Each layer of the CNN block is composed of 3 × 3 convolution (Conv), batch normalization (BN), and rectified linear unit (ReLU) operations. In fact, this CNN block structure is the one that has been proven to be effective in network training by He et al. [14].

Similar to the U-Net, the pixelwise cross entropy is used as the loss function of the network, as defined in

(1) $$\begin{array}{c} E=\underset{x}{\sum }\log\left(p_{l\left(x\right)}\left(x\right)\right), \end{array}$$

where *l* is the true label of each pixel and *p*_*k*_(*x*) is the softmax of pixel *x* in the output feature map, which is defined as

(2) $$\begin{array}{c} p_{k}\left(x\right)=\frac{\exp\left(a_{k}\left(x\right)\right)}{\sum_{k^{\prime }}^{K}\exp\left(a_{k^{\prime }}\left(x\right)\right)}, \end{array}$$

where *a*_*k*_(*x*) denotes the activation in feature channel *k* of pixel *x* and *K* is the number of classes.

The network is trained using the MITOS2012 dataset [27] which has pixel-level strong labels. Input images and their corresponding segmentation maps are fed into the network for training. The trained network performs an end-to-end prediction, and the output feature map shares the same width and height as those of the input images. The output feature map indicates a probability of a pixel that it belongs to mitosis.

After getting the segmented mitosis, the minimum circumscribed rectangle is labeled as the bounding box of mitosis, which will be taken as the ground truth. In this paper, if the weak label (a point labeled at the center of the mitotic nucleus) is within the marked bounding box, the sample will be taken as positive.  Figure 3 shows some examples of the labeled bounding boxes.

### 3.2. Mitosis Detection

After generating strong labels, the R-CNN [21] algorithm is employed for mitosis detection. R-CNN has been a representative and powerful CNN-based object detection method since recent years. R-CNN performs a four-step detection routine, i.e., region proposal generation, CNN-based feature extraction, SVM-based region classification, and bounding box regression. A selective search algorithm is employed to generate region proposals, which will be fed into a CNN to extract features after region wrapping. During the training phase, the generated bounding boxes in Section 3.1 are used as the ground truth. 32 positive samples and 96 negative samples are composed together as a minibatch, which is consistent to the original R-CNN, and are proven to be an optimized combination. It should be noticed that theoretically any object detection method can be employed here, and more powerful object detection method may obtain more accurate results.

## 4. Experimental Results

### 4.1. Datasets

In the experiments, three mostly used datasets for mitosis detection are employed, i.e., AMIDA2013 [12], ICPR2014 [28], and TUPAC2016 [29]. All these datasets contains H&E-stained breast cancer histopathological section view.  Figure 4 shows some exemplars from the datasets.

The AMIDA2013 dataset consists of 1083 samples from 23 volunteers, and each volunteer has at least 10 views with dimension of 2000 × 2000 and resolution of 0.25 pixels/*μ*m. Images from the AMIDA2013 dataset are obtained by Aperio Scanscope XT slice scanner. Images are labeled by experts from University Medical Center Utrecht, and each view is labeled by two experts independently. For the AMIDA2013 dataset, 550 samples of 12 volunteers are taken as the training set and others as the validation set.

The ICPR2014 dataset was firstly proposed for the ICPR2014 mitosis detection competition. It is composed of two subsets of images scanned by Aperio Scanscope XT and Hamamatsu Nanozoomer 2.0-HT digital slice scanner, respectively. The dimension of images from this dataset is 1539 × 1376 and the resolution is 0.2455 pixels/*μ*m. The dataset is labeled by two pathologists independently, and 749 mitosis are labeled out of 1200 views from 11 volunteers. In this paper, 816 views are selected as the training set, and 96 are taken as the validation data, which is consistent with Ref. [18] and Ref. [20].

The TUPAC2016 dataset consists of two parts. The first part contains samples from 23 volunteers, and this part is the same as the AMIDA2013 dataset. The second part contains samples from 50 volunteers with dimension of 5657 × 5657, which are scanned using Leica SCN 400 digital slice scanner. Each image is labeled by two pathologists independently. In the experiment, validation samples are selected by every 7 volunteers from volunteer no.30, and the others are taken as training samples. This strategy is consistent with Ref. [18].

### 4.2. Evaluation Metrics

Evaluation is performed according to the ICPR2014 contest criteria. A detected mitosis is counted as correct if its center point is localized within a range of 8 *μ*m from its ground truth. Here, the center point of detected mitosis is defined as the diagonal intersection of its bounding box. Three metrics, namely, precision, recall, and *F*_1_-score are employed as the quantitative indicators, which are defined in

(3) $$\begin{array}{c} \text{Precision}=\frac{\text{TP}}{\text{TP}+\text{FP}},\\ \text{Recall}=\frac{\text{TP}}{\text{TP}+\text{FN}},\\ F_{1}‐score=\frac{2\times \text{Recall}\times \text{Precision}}{\text{Recall}+\text{Precision}}, \end{array}$$

where TP is the number of true mitosis which are detected, FP is the number of falsely detected mitosis, and FN is the number of true mitosis which are not detected. Precision indicates how many true mitosis are detected out of all the detected instances. Recall indicates how many true mitosis are detected out of all mitosis. *F*_1_-score gives a comprehensive combination of Precision and Recall.

### 4.3. Implementation Details

The experiments are carried out on a computer with Intel Core i7 CPU, Nvidia GTX 2080Ti GPU, and 16 GB RAM. All the codes are implemented using Python 3.6 as the programming language and PyTorch 1.9.0 as the deep learning framework. Both networks are trained 100 epochs with Adam optimizer and batch size of 8. During training, the learning rate is initialized as 10^−3^ and decreased to 10^−6^ after 100 epochs.

### 4.4. Results and Comparisons

Detection results and comparisons with some state-of-the-art methods considering the three criteria are listed in Table 1. It should be noticed that all the results of the referred methods are reported by the literatures. Some visual results are shown in Figure 5. In Figure 5, rectangles indicate the bounding boxes of detected mitosis, and dot marks indicate the ground truth label (enlarged for visual effect).

From the results, we can see that the proposed method achieves the best results compared with the referred methods in most of the cases. Li et al.'s method [18] is a CNN-based mitosis detection method which uses two concentric circles to label a mitosis area. The proposed method outperforms Li et al.'s method on all the three considered datasets with respect to most of the criteria. Since the proposed method employs a segmentation network to generate strong labels, the detection network can be better trained with this more adequate training data, and thus, more competent prediction performance is obtained. The IDSIA [12] method employs a multicolumn max pooling convolutional neural network (MCMPCNN) for supervised pixel classification. However, only weak labels are used in its network training, which influences the prediction ability of IDSIA.

### 4.5. Impact of Label Generation

To further corroborate the effectiveness of the label generation strategy used in this paper, an additional experiment is performed on the TUPAC2016 dataset, and the results are listed in Table 2, in which Manual means the bounding boxes of mitosis are marked manually, i.e., the minimum rectangle that can surround the mitosis and include the ground truth point, U-Net means the mitosis is segmented using the original U-Net network [25], and Proposed means the mitosis is segmented using the proposed segmentation network.

From the results, we can see that labels generated by the proposed segmentation network are slightly better than the original U-Net, which can be attributed to the fact that the proposed network can provide a more accurate pixel class prediction and thus provide a more accurate bounding box. However, different segmentation methods have similar final detection results, and they are also similar with that of manual labeling. We can conclude that segmentation-based label generation is beneficial to mitosis detection with nearly no accuracy loss.

## 5. Conclusions

In this paper, a deep learning-based method for mitosis detection in breast histopathology images is proposed. The method is aimed at solving the problem of the insufficiency of strongly labeled samples by incorporating a bounding box label generation process before mitosis detection. Experimental results show that the proposed label generation strategy can promote the mitosis detection performance in a large extent. The main limitation of the proposed method is that the employed object detection method R-CNN needs a long time of training, although it can be solved by integrating a more powerful object detection method into the proposed detection routine.

## Figures and Tables

**Figure 1:** Flowchart of the proposed method.

**Figure 2:** Architecture of the segmentation network.

**Figure 3:** Examples of labeled bounding boxes. (A) Original. (B) Original with mask. (C) Original with bounding box. (a, b) True positives. (c, d) False positives.

**Figure 4:** Exemplars from the datasets: (a) AMIDA2013, (b) ICPR2014, and (c) TUPAC2016.

**Figure 5:** Some detection results. Rectangles indicate the bounding boxes of detected mitosis, and dot marks indicate the ground truth label (enlarged for visual effect): (a) AMIDA2013, (b) ICPR2014, and (c) TUPAC2016.

**Table 1:** Detection results.

Datasets	Methods	Recall	Precision	*F*_1_-score
AMIDA2013	IDSIA [12]	0.612	0.610	0.611
	Li et al. [18]	0.677	0.669	0.673
	Proposed	0.689	0.690	0.689
ICPR2014	Yancey et al. [20]	—	—	0.507
	Li et al. [18]	0.682	0.541	0.603
	Proposed	0.733	0.539	0.621
TUPAC2016	Li et al. [18]	—	—	0.717
	Proposed	0.766	0.843	0.803

**Table 2:** Detection results.

Label generation method	Recall	Precision	*F*_1_-score
Proposed	0.766	0.843	0.803
U-Net	0.751	0.840	0.793
Manual	0.779	0.850	0.813

## Data Availability

The data used to support the findings of this study are all publicly available datasets deposited in the following websites: (1) AMIDA2013 dataset, https://tupac.grand-challenge.org/Dataset/. The AMIDA2013 dataset is contained as part of the TUPAC2016 dataset (also declared in the manuscript). These two datasets are publish by the same organization, so the AMIDA2013 dataset cannot be accessed as its own. Anyone can get the AMIDA2013 dataset through downloading the TUPAD2016 dataset. Please refer to [29]. (2) ICPR2014 dataset,https://mitos-atypia-14.grand-challenge.org/Dataset/. (3) TUPAC2016 dataset,https://tupac.grand-challenge.org/Dataset/. (4) MITOS2012 dataset, http://www.icpr2012.org/contests.html
